# The Role of 12/15-Lipoxygenase and Its Various Metabolites Generated from Multiple Polyunsaturated Fatty Acids as Substrates in Inflammatory Responses

This article has been retracted.

**DOI:** 10.1155/2022/4589191

**Published:** 2022-09-25

**Authors:** Ruyu Tan, Bing Yan, Chengshuo Wang, Luo Zhang

**Affiliations:** ^1^Department of Otolaryngology Head and Neck Surgery, Beijing TongRen Hospital, Capital Medical University, Beijing 100730, China; ^2^Beijing Key Laboratory of Nasal Diseases, Beijing Institute of Otolaryngology, Beijing 100005, China

## Abstract

12/15-lipoxygenase (12/15-LOX) is a member of the lipoxygenase family, which can catalyze a variety of polyunsaturated fatty acids (PUFA) to produce different metabolites, such as 12-hydroxyeicosatetraenoic acid (12-HETE), 15-HETE, lipoxin (LX), hepoxilin, resolvin, protectin, and maresins. 12/15-LOX and its metabolites take part in inflammatory responses and mediate related signalling pathways, playing an essential role in various inflammatory diseases. So the definition, catalytic substrates, metabolites of 12/15-lipoxygenase, and their roles in inflammatory responses are reviewed in this article.

## 1. Introduction

The discovery of lipoxygenase has a long history; its naming and classification are also various. At the same time, the definition of lipoxygenase is more complicated and ambiguous because of the differences in lipoxygenase (LOX) in Homo sapiens, mice, rabbits, and other organisms. Therefore, this article reviews the discovery history of LOX, the different terminology, the differences of LOX in other species, and the definition of 12/15-LOX.

The classification of fatty acids is complex, and the metabolites produced by 12/15-LOX catalyzed by different substrates are also diverse. Therefore, this article reviews the definition, classification of polyunsaturated fatty acids (PUFA), and the other metabolites produced by *ω*-3 and *ω*-6 fatty acids catalyzed by 12/15-LOX, such as 12-hydroxy-eicosatetraenoic acid (12-HETE), 15-HETE, lipoxin (LX), hepoxilin, resolvin, protectin, and maresins. This article reviewed the role of the above metabolites in the inflammatory response.

## 2. Classification and Formation of Polyunsaturated Fatty Acids

Fatty acid (FA) is the crucial component of lipids, which can be divided into saturated fatty acid, monounsaturated fatty acid, and polyunsaturated fatty acid (PUFA). PUFA refers to straight-chain fatty acids with more than two double bonds and a carbon chain length of 18-22 carbon atoms, which can be divided into *ω*-3, 6, 7, and 9 fatty acids. This article mainly discusses the various metabolites generated from *ω*-3 and *ω*-6 as substrates.

*ω*-3 fatty acids mainly contain *α*-linolenic acid (ALA), docosahexaenoic acid (DHA), and eicosapentemacnioc acid (EPA). ALA is a precursor for the production of DHA and EPA. *ω*-6 fatty acids mainly contain linoleic acid (LA), gamma-linolenic acid (GLA), dohomo-gamma-linolenic acid (DGLA), and arachidonic acid (AA). GLA can be converted from linoleic acid or linolenic acid in vivo [1].

Arachidonic acid has 20 carbon atoms and four double bonds. It is the most abundant polyunsaturated fatty acid in mammals, accounting for about 40-50% of the total polyunsaturated fatty acids in the human body. In some nervous tissues, the content of arachidonic acid can even reach 70% [1]. A tiny amount of arachidonic acid exists in the cytoplasm and extracellular fluid in an active free state. Most of the arachidonic acid exists in the phospholipids of the cell membrane in an inactive esterified state and can be catalyzed by cytoplasmic phospholipase A2 (cPLA2) to generate arachidonic acid. There are two primary sources of arachidonic acid in the human body. One is directly absorbed in the human intestinal tract through diet. The second is that linoleic acid generates GLA through dehydrodesaturation in the human body. GLA generates eicosatrienoic acid by extending the carbon chain, and eicosatrienoic acid causes eicosatrienoic acid through desaturation, namely, arachidonic acid. Dietary supplements can only supplement linoleic acid, and the human body cannot synthesize it alone. Therefore, the *ω*-3 fatty acids with ALA as the parent and the *ω*-6 fatty acids with LA as the parent are both essential fatty acids for the human body (Figure 1).

## 3. Classification and Naming of LOX

Lipoxygenase (LOX) can catalyze a variety of polyunsaturated fatty acids, generate different metabolites, and participate in many different physiological or pathological processes, such as inflammatory responses. LOX is widely found in eukaryotes such as plants [1], animals [2], and fungi [3]. LOX is nonheme ferritin that binds two calcium ions and has a catalytic center containing iron ions. It consists of a single polypeptide chain with an N-terminal domain and a terminal C-active center domain. The former regulates the binding of enzymes to substrates, and the latter is responsible for catalysis [1].

In plants, LOX mainly uses linolenic acid and LA as substrates [4] and participates in plant growth, development, and senescence [1]. In animals, LOX mainly uses AA as a substrate [5] to generate a series of eicosanoids, which are involved in forming an inflammatory response, immune response, and related signalling molecules [2]. Therefore, LOX is also often referred to as “ALOX”, that is, arachidonic acid lipoxygenase (ALOX), which catalyzes the reaction of arachidonic acid. The gene encoding lipoxygenase has also been found in some prokaryotes, such as in 38 Gram-negative bacteria [6].

The discovery of LOX has a long history, and as the understanding of LOX deepens, the naming and classification become more complicated. First, according to the position of the oxygen molecule inserted in the oxidation of AA, it can be divided into 5-LOX, 8-LOX, 11-LOX, 12-LOX and 15-LOX. For example, LOX that catalyzes the oxidation of the 12th carbon atom of the fatty acid hydrocarbon backbone is called “12-LOX” [1]. Secondly, in space, when the connected groups are different, the carbon atoms are arranged chiral so that they can be divided into R and S configurations, such as 12-LOX can be divided into 12R-LOX and 12S-LOX. Finally, the different primary expressing cells can be divided into epidermal, reticulocyte, leukocyte, and platelet types. For example, 12S-Lox in mice can be further divided into epidermal 12S-Lox, leukocyte-type 12S-Lox, and platelet-type 12S-Lox.

Six different isoforms of Lox can be found in mice [2], namely, 5S-Lox, leukocyte-type 12S-Lox, platelet-type 12S-Lox, epidermal 12S-Lox, epidermal 12R-Lox, and epidermal 8R-Lox. In Homo sapiens, five different LOX isoforms can be found, namely, 5S-LOX, reticulocyte-type 15S-LOX, platelet-type 12S-LOX, epidermal 12R-10X, and epidermal 15S-LOX [5, 7].

Different types of LOX from other species can be similar in the specificity of substrates or significantly different, thus showing the characteristics of various enzymes. Judging from the similarity of amino acid sequences, 5-LOX of mice and 5-LOX of Homo sapiens have high amino acid sequence similarity. Both are involved in the synthesis of leukotrienes in mammals. The platelet-type 12S-LOX of mice and the platelet-type 12S-LOX of Homo sapiens also have high amino acid sequence similarity. The enzyme is mainly distributed in platelets in normal tissues and can also be detected in various tumor tissues. The metabolite 12S-hydroxyeicosatetraenoic (12S-HETE) produced by AA has also been shown to be involved in tumor angiogenesis [8], cell proliferation, and apoptosis and is closely related to tumor occurrence, development, and metastasis. The amino acid sequences of mice epidermis 12R-Lox, mice epidermis 8R-Lox, human epidermis 12R-10X, and human epidermis 15S-LOX are very similar. Human epidermal 15S-LOX is encoded by the ALOX15B gene [9] and is mainly expressed in skin and other epithelial cells [10], also often referred to as 15-LOX-2.

## 4. Definition of 12/15-LOX

According to the specificity of the enzymes, the leukocyte-type 12S-LOX and the reticulocyte-type 15S-LOX of different species can be divided into a class, collectively referred to as “12/15-LOX”, or “12S/15S-LOX”, which includes leukocyte-type 12S-LOX of mice, leukocyte-type 12S-LOX of rabbits, reticulocyte-type 15S-LOX of rabbits, and human reticulocyte-type 15S-LOX. The definition of this concept is related to the history of LOX discovery. The LOX enzyme in mammals was first detected in rabbit reticulocytes in 1975, called reticulocyte type 15S-LOX. This enzyme is involved in the maturation and differentiation of reticulocytes. Later, leukocyte-type 12S-LOX was found in rabbit leukocytes, which had 99% similarity at amino acid level with rabbit reticulocyte-type 15S-LOX. At the same time, these two kinds of LOX of rabbits have high similarity in amino acid levels with the leukocyte type 12S-lox of mice and the human reticulocyte type 15S-LOX. Therefore, these enzymes are collectively referred to as “12/15-LOX” [8].

Human reticulocyte-type 15S-LOX is a critical enzyme in human lipid metabolism. This enzyme, which is also the main content of this paper, is mainly expressed in immune cells and is encoded by the ALOX15 gene [9]. Because the enzyme was found initially in reticulocytes [10] and is abundantly expressed in immature reticulocytes that arise from repeated bleeding or anemia [8, 11, 12], it is called reticulocyte-type 15S-LOX or 15-LOX-1. The amino acid sequences of 15-LOX-1 and 15-LOX-2 are only 40% similar [13], and their biological functions are very different [14]. 15-LOX-1 can catalyze various PUFA reactions such as arachidonic acid, linolenic acid, and linoleic acid [1], which can not only produce a series of inflammatory mediators to promote the occurrence and development of inflammation but also produce a series of specialized proresolving mediators (SPMs) [15], such as lipoxin, resolvin, protectin, and maresins. SPMs can inhibit the development of inflammation.

## 5. Metabolites Using Arachidonic Acid as Substrates and their Roles in Inflammation

Arachidonic acid is an essential fatty acid involved in human growth and development. On the one hand, arachidonic acid can provide ATP as a direct energy source in the body through *β*-oxidation. On the other hand, arachidonic acid can also generate a series of eicosanoids. Arachidonic acid has three main metabolic pathways in the human body, and it can generate prostaglandins and thromboxanes through cyclooxygenase (COX). Arachidonic acid can also create leukotrienes, 12-HETE, 15-HETE, lipoxin, hepoxilin, and other compounds through LOX. Arachidonic acid can also be catalyzed by cytochrome P450 monooxygenase (CYP450) to generate epoxyeicosatrienoic acids (EETs) (Figure 2).

### 5.1. Product 12S-HETE

Arachidonic acid can generate a mixture of 12S-hydroperoxy-eicosatetraenoic acid (12S-HpETE) and 15S-HpETE under the action of 12/15-LOX [16]. 12S-HpETE is unstable and can continue to develop 12S-HETE under the catalysis of phospholipid-hydroperoxide glutathione peroxidase (phGPx), or it can be spontaneously reduced to 12S-HETE without enzymatic catalysis.

12S-HETE is a proinflammatory mediator, and it can promote the expression of Rho-associated kinase (ROCK), thereby activating the nuclear factor *κ*-B (NF-*κ*B) signalling pathway, increasing the expression of intercellular adhesion molecule-1 (ICAM-1), and promoting mononuclear adhesion of cells to the endothelium [17]. NF-*κ*B can also regulate the expression of monocyte chemotactic protein 1 (MCP-1) in endothelial cells and promote monocyte adhesion to endothelial cells, which indicates that MCP-1 is also held by 12S-HETE [18].

### 5.2. Product 15S-HETE

In both airway epithelial cells and eosinophils, a large amount of 15-LOX-1 can catalyze the production of 15S-HpETE from AA. Like 12S-HPETE, 15S-HpETE is also unstable and can be catalyzed by phGPx to generate 15S-HETE or degraded to 15S-HETE without enzymatic catalysis [16].

15S-HETE regulates the function of vascular smooth muscle and endothelial cells. Under hypoxic conditions, 15-LOX-1 was induced to produce large amounts of 15S-HETE. High concentrations of 15S-HETE (10–30 *μ*M) can activate intracellular peroxisome proliferator-activated receptors *γ* (PPAR*γ*), regulate metabolic processes, and enhance the expression of macrophage surface scavenger receptors. Thus, it can improve the phagocytosis of macrophages, regulate lipid metabolism [19], exert an anti-inflammatory effect, and promote the resolution of inflammation.

At the same time, 15S-HETE can also induce tyrosine phosphorylation of EGF receptors in vascular smooth muscle cells, increase the expression of STAT3-dependent MCP-1, and promote the proliferation and migration of vascular smooth muscle cells to the intima [19]. 15S-HETE can also increase the tyrosine phosphorylation of the intercellular tight junction protein ZO-2 through the Pyk2/Src signalling pathway, disrupting its connection with claudin-1 and claudin-5 and disrupting endothelial cell barrier function. This can lead to endothelial cell dysfunction [20], promote the migration of neutrophils and mast cells into the tracheal lumen, promote mucus secretion, and aggravate the inflammatory response.

### 5.3. Product Lipoxin

Lipoxins are often referred to as “brake signals” in the inflammatory response. Because of its apparent anti-inflammatory effect [21, 22], it plays a vital role in the body's inflammation. Lipoxins contain three hydroxyl groups and four conjugated double bonds. The hydroxyl position and carbon atom conformation can be divided into lipoxin A4 (LXA4) and LXB4 and their isomers 15-epimer-lipoxin A4 (15-epi-LXA4) and 15-epi-LXB4. LXA4 has the most potent anti-inflammatory effect (Figure 3).

Lipoxins are synthesized sequentially from multiple LOXs in different cells. There are three main synthetic routes. The first route is mainly in the mucosal tissue of the respiratory tract. Arachidonic acid in eosinophils, epithelial cells, and monocyte-macrophages is catalyzed by 15-LOX-1 to generate the labile intermediate 15S-HpETE. 15S-HpETE can not only be degraded to 15S-HETE but also be catalyzed by 5-LOX in neighboring polymorphonuclear leukocytes (PMN) to generate lipoxin. 15S-HpETE can synthesize the anti-inflammatory mediator lipoxin and reduce the synthesis of the proinflammatory mediator leukotrienes by competing with the critical enzyme 5-LOX, thereby exerting a powerful anti-inflammatory effect. The second pathway is mainly in the vascular endothelium. Arachidonic acid is first catalyzed by 5-LOX in leukocytes to generate leukotriene A4 (LTA4). LTA4 is then catalyzed by 12-LOX in platelets to generate LXA4 and LXB4. The third route has to do with aspirin. AA is also catalyzed by aspirin-acetylated COX-2 and 5-LOX in leukocytes to generate 15-epi-LXA4 and 15-epi-LXB4 (Figure 4).

There are three central lipoxin receptors: lipoxin A4 receptor (ALX), cysteine leukotriene receptor (CysLTR), and intracellular aryl hydrocarbon receptors. ALX is a transmembrane G protein-coupled receptor and the primary lipoxin receptor, expressed in PMNs, macrophages, and epithelial cells. In macrophages, LXA4 can enhance the activity of its surface receptor CD36, thereby enhancing the recognition of apoptotic PMNs by macrophages, enhancing their ability to phagocytose PMNs [23], inhibiting the activation of NF-*κ*B, inhibiting proinflammatory medium expression, and reducing the release of proinflammatory factors MCP-1 and IL-8 during its phagocytosis [24, 25].

In PMNs, ALX binds to LXA4, inhibits the chemotaxis of PMNs to inflammatory sites, inhibits the adhesion between neutrophils and endothelial cells and epithelial cells, and reduces the infiltration of neutrophils. In a mice back inflammation model [21], a peak of PMN recruitment first appeared during the peak period of the inflammation, and later with the subsidence of the inflammatory response, an elevation of LXA4 expression seemed again.

CysLTR and ALX have certain homology. LXA4 can bind to ALX and competitively bind CysLTR with LTC4 and LTD4 of the leukotriene family. Through this competitive inhibition, LXA4 can antagonize the proinflammatory effects of leukotrienes, thereby exerting an anti-inflammatory influence.

### 5.4. Product-Hepoxilins (HXs)/Trioxilins (TrXs)

Arachidonic acid is catalytically metabolized to 12S-HpETE by 12S-LOX. 12-HpETE can be catalyzed by phGPx to generate 12S-HETE and can also be isomerized into biologically active hepoxilin A3 (HXA3) and biologically inactive HXB3. HXA3 and HXB3 can then generate trioxilin A3 (TrXA3) and TrXB3 through epoxide hydrolase (EH) [26].

The naturally occurring HXs in the human body are chemically and biologically unstable. At the same dose, stable TrXs showed no biological activity. HXs can participate in various physiological processes such as releasing inflammatory mediators, insulin secretion, calcium regulation, potassium regulation, and cell volume regulation [26]. HXA3 is also a chemokine for human neutrophils, which recruits neutrophils to injured sites by rapidly releasing calcium ions in neutrophils, promoting neutrophil chemotaxis, and increasing vascular permeability. HXA3 leads to the generation of early signals of the inflammatory response. In some inflammatory diseases such as pneumonia, infection of respiratory epithelial cells can induce the production of HXA3, which promotes the entry of neutrophils into the airways [27]. Then, neutrophils can synthesize and release histamine, leading to airway inflammation. Neutrophils have two modes of sterilization and can directly phagocytose pathogens to kill bacteria. Neutrophils can also encapsulate and destroy invading pathogens through a novel form of death distinct from necrosis and apoptosis, releasing a network of DNA and various enzymes called neutrophil extracellular traps (NETs). The process by which neutrophils release NETs is called NETosis [28], and HXA3 can directly induce this NETosis [29].

## 6. Metabolites Using Linoleic Acid (LA) as Substrates and their Roles in Inflammation

Linoleic acid and arachidonic acid are both *ω*-6 PUFAs, which are PUFAs containing 18 carbon atoms and two cis double bonds. Firstly, linoleic acid can generate *γ*-linolenic acid (GLA) through dehydrodesaturation in the human body. GLA generates eicosatrienoic acid by extending the carbon chain. Eicosatrienoic acid is then desaturated to form eicosatetraenoic acid, also known as arachidonic acid. Secondly, linoleic acid can be directly oxidized by 15-LOX to volatile hydroperoxy-octadecadienoic acid (HpODE). HpODE can be catalyzed by phGPx or now degrade itself to form stable hydroxyoctadecadienoic acid (HODE). The HODEs are mainly 9S-HODE and 13S-HODE [30] (Figure 5).

HODE is secreted in macrophages, endothelial cells, platelets, and smooth muscle cells. HODE can play multiple roles in signalling and regulating inflammation by acting as a ligand for PPAR*γ* and G protein-coupled receptor 132 (GPR132).

9S-HODE and 13S-HODE are ligands for the type 2 nuclear receptor peroxisome proliferators-activated receptors *γ* (PPAR*γ*), which can activate the PPAR*γ* signalling pathway [31]. The transcriptional activity of PPAR*γ* can be induced by arachidonic acid and 15S-HETE. However, as endogenous ligands, 9S-HODE and 13S-HODE appear to be more effective in influencing and inducing the transcriptional activity of PPAR*γ*. So 9S-HODE and 13S-HODE can inhibit the activation of the NF-*κ*B signalling pathway, inhibit leukocyte aggregation, inhibit airway inflammation, reduce mucus secretion, and reduce inflammatory markers production [32], which has an anti-inflammatory effect. PPAR*γ* is expressed in both monocyte-macrophages and foam cells. Both 9S-HODE and 13S-HODE can inhibit the proliferation of monocytes. 9S-HODE can induce apoptosis. 13S-HODE can make the cell cycle stay in the S phase. The production of various inflammatory cytokines in monocytes-macrophages can also be inhibited by 9S-HODE and 13S-HODE, such as TNF-*α*, IL-1*β*, and IL-6, thereby inhibiting the migration and inflammatory response of monocytes. CC chemokine receptor (CCR2) can mediate the aggregation of monocytes on the blood vessel wall. 9S-HODE and 13S-HODE can also inhibit the expression of CCR2, reduce the chemotaxis of monocytes, and inhibit atherosclerosis. But at the same time, 9S-HODE and 13S-HODE can activate PPAR*γ*, promote the differentiation of monocytes into M2 macrophages with an anti-inflammatory effect, and induce the expression of scavenger surface receptor CD36, thereby enhancing the phagocytosis of macrophages, and increase the risk of inflammation and atherosclerosis [30].

In the early stage of atherosclerosis, 13S-HODE can promote the apoptosis of monocytes and macrophages, reduce cellular structural damage, and delay disease progression. But at a later stage, elevated 13S-HODE promotes apoptosis in many macrophages, and the apoptotic cells exceed the body's clearance capacity, which may, in turn, encourage plaque rupture, thrombosis, and disease progression. 9S-HODE and 13S-HODE also increased the expression of the fatty acid-binding protein (FABP) in macrophages. FABP mainly exists in adipose tissue and macrophages. It is a peripheral membrane protein that promotes fatty acid transport and plays an essential role in regulating fatty acid metabolism and inflammatory responses. Overexpression of FABP in macrophages can cause excessive deposition of triglycerides and cholesterol to form foam cells, leading to atherosclerosis [33].

9S-HODE is also a high-affinity ligand of GPR132 and has proinflammatory effects, but 13S-HODE is not a ligand of GPR132. GPR132 is strongly expressed in macrophages and is a class of proinflammatory substances produced by lipoprotein-associated phospholipase A2 (Lp-PLA2) secreted by macrophages in the vascular intima after hydrolysis and oxidation of phospholipids in low-density lipoprotein. It can regulate cell chemotaxis, cause abnormal endothelial function, stimulate the production of various adhesion factors, further chemotactic inflammatory cells, and enhance inflammatory response [33].

## 7. Metabolites Using EPA and DHA as Substrates and their Roles in Inflammation

There are two isomers of linolenic acid, *α*-linolenic acid (ALA) and GLA. ALA is a kind of octadecatrienoic acid containing three cis double bonds, has strong reducibility, and is readily oxidized by high temperature, ultraviolet light, oxygen, and heavy metal ions. ALA can generate eicosapntemacnioc acid (EPA) through desaturation, carbon chain elongation, and desaturation. EPA can in turn generate DHA through the elongation and desaturation of carbon chain (Figure 6).

### 7.1. Anti-Inflammatory Effects of EPA and DHA

EPA is unstable in nature and easy to oxidize and crack. It has a variety of physiological functions, such as anti-platelet aggregation, preventing thrombosis, improving blood lipid disorders, improving body resistance, anti-inflammatory, and inhibiting tumor cell proliferation. DHA also exerts the effects of being anti-inflammatory and neuroprotective. EPA and DHA's physiological and anti-inflammatory functions are closely related to their proportions on the cell membrane. The ratio of EPA to DHA on immune cell membranes in Western humans is approximately 1 : 2.5 [34], and this content can be altered by diet. EPA and DHA enhance the fluidity of the cell membrane, thereby affecting the ion channels and receptors of the cell membrane, reducing the production of IL-6 and IL-8 by vascular endothelial cells, and reducing the production of IL-1*β*, TNF-*α*, reducing the expression of macrophage adhesion molecules intercellular adhesion molecule-1 (ICAM-1) and VCAM-1, reducing the adhesion of monocytes and macrophages, and inhibiting intracellular signal transduction [35]. Therefore, eating foods rich in EPA and DHA, such as deep-sea fish, can reduce the content of arachidonic acid on the cell membrane and affect the inflammatory response involved in arachidonic acid [36].

EPA can generate prostaglandins through the COX pathway. EPA can also be catalyzed by 5-LOX to generate leukotrienes or by 12-LOX to generate 12-hydroxyeicosapentaenoic acid (12-HEPE) and hepoxilin B4 (HXB4). HXB4 can be further catalyzed by epoxy hydrolase (EH) to generate trioxilin B4 (TrXB4). EPA can also be catalyzed by 15-LOX to generate 15-HEPE, lipoxin A5 (LXA5), or LXB5. DHA can be catalyzed by 11/12-LOX to generate 14-hydroperoxydocosahexaenoic acid (14-HpDoHE), which is further catalyzed to generate Maresin 1 (MaR-1), 14-hydroxydocosahexaenoic acid (14-HDoHE), and HXB5. EH can further catalyze HXB5 to generate TrXB5 (Figure 7).

The anti-inflammatory effects of both of them are mainly by activating the PPAR pathway as ligands and inhibiting the NF-*κ*B pathway. Both DHA and EPA can start PPAR but have the strongest affinity with PPAR*α*, which can activate PPAR*α* to enter cells and promote the synthesis of the inhibitory protein I*κ*B of dimer NF-*κ*B. Therefore, the phosphorylation of I*κ*B by I*κ*B kinase (IKK) is reduced, resulting in the inability of NF-*κ*B to dissociate from I*κ*B. Thus, the subunit p65 of dimeric NF-*κ*B cannot be transferred into the nucleus and cannot bind to specific proteins on DNA, which reduces the transcription of inflammatory factor-related genes. Therefore, it reduces the production of inflammatory cytokines TNF-*α*, IL-1*β*, and IL-6 and reduces the expression of adhesion molecules ICAM-1 and VCAM-1 [37]. EPA can also inhibit the MAPK activity of the downstream signalling pathway after the binding of LPS to its Toll-like receptor, affect the MAPK signal transduction in macrophages, further reduce the phosphorylation of I*κ*B, and inhibit the NF*κ*B signalling pathway. EPA and DHA can also bind to the G-protein-coupled receptor GPR120, which is highly expressed in adipocytes and macrophages, to enhance its signal transduction and maintain I*κ*B levels in the cytoplasm, thereby inhibiting NF*κ*B activation [36].

### 7.2. Competitive Inhibition of AA by EPA and DHA

*ω*-3 and *ω*-6 fatty acids are essential components of cell membranes. The relative balance of these two fatty acids, as well as the relative balance of their metabolites, eicosanoids, is the fundamental factor in maintaining body health and is also one of the most important mechanisms for the actions of EPA and DHA. The metabolic competition of *ω*-3 and *ω*-6 fatty acids is mainly the metabolic competition of DHA, EPA, and AA, especially the metabolic competition of EPA and AA.

The competitive inhibition of EPA synthesized by ALA and AA synthesized by LA is mainly reflected in the competitive binding of COX and LOX. Although their metabolites are not identical, their metabolic pathways are similar. They are all precursors for the synthesis of 20-carbon fatty acid derivatives. They can both synthesize PGs through the COX pathway or synthesize LTs through the 5-LOX pathway. The derivative product of AA has intense activity, and the derivative product of EPA has weak activity. Therefore, the ratio of EPA to AA affects the severity of the inflammatory response. The higher the EPA content, the weaker the inflammatory response. The higher the content of AA, the more inadequate the inflammatory response.

AA synthesizes PGD2, PGE2, PGF2, and PGI2 in the COX pathway. EPA and AA have similar chemical structures, so COX enzymes can catalyze EPA to generate PGD3, PGE3, PGF3, and PGI3 through competitive inhibition. By competing with metabolic enzymes, EPA reduces the amount of PGs and TXs produced by AA and exerts an anti-inflammatory effect. The derivatives of EPA and AA are structurally similar and have the same metabolic pathway. When they coexist, they are the substrates for the competitive inhibition of their respective metabolic enzymes, resulting in competitive inhibition (Figure 8(a)). DHA is not a precursor fatty acid of mammalian prostaglandins. Although DHA cannot generate PGs through metabolism, DHA can also bind to COX-2, thereby inhibiting the production of PGs, TXs, and LTs in the AA metabolic pathway. PGI3 produced by EPA in vascular tissue can inhibit platelet aggregation, while TXA3 produced by EPA in platelets does not have the effect of TXA2 on promoting vasoconstriction and platelet aggregation [38].

AA can be metabolized in the LOX pathway to generate LTB4, LTC4, LTD4, and LTE4. EPA can also be catalyzed by LOX to generate LTB5, LTC5, LTD5, and LTE5. The structures of their derivatives are similar, the LOX metabolic pathways are similar, and the metabolic sites are also in leukocytes, which are competitive inhibition of each other [38] (Figure 8(b)).

### 7.3. Product Resolvin and Protectin

Resolvin (Rv) and protectin (PD) which derived from EPA and DHA are decisive inflammatory self-limiting factors with substantial anti-inflammatory effects (Figure 9). The enzymes which involved in the synthesis of resolvin and protectin are 5-LOX, 15-LOX, and COX-2 acetylated by aspirin. Resolvin derived from EPA, called RvE, and resolvin derived from DHA, called RvD, can attenuate NF*κ*B signalling activation [39]. The protective effect of DHA on nerve cells is also related to its metabolite protectin, which can prevent nerve cell necrosis and promote the repair and regeneration of injured nerve cells.

Resolvin is produced through multiple transcellular pathways. DHA can be catalyzed by 15-LOX to generate 17S-hydroperoxy-docosahexaenoic acid (17S-Hp-DHA) and then catalyzed by 5-LOX to generate Resolvin D1(RvD1), RvD2, RvD3, and RvD4. DHA can also develop 17R-RvD, also known as AT-RvD1, AT-RvD2, AT-RvD3, and AT-RvD4, by acetylated COX-2 in endothelial cells and 5-LOX in leukocytes in the presence of aspirin [40]. EPA can also be catalyzed by aspirin-acetylated COX-2 to generate 18R-HpETE and then by 5-LOX in leukocytes to generate Resolvin E1 (RvE1) and RvE2 [40] (Figure 10).

Protectin is also derived from the product of DHA catalyzed by lipoxygenase [40]. At the site of inflammation, DHA is first catalyzed by 15-LOX to 17S-Hp-DHA, then converted to epoxide intermediate by COX, and then enzymatically hydrolyzed to generate biologically active ProtectinD1 (PD1) [41]. PD1 has anti-inflammatory effects [42]. PD1 also protects nerves when it is produced in the nervous system, so it is also called neuroprotectinD1 (NPD1). There are six isomers of PD1, but none of the isomers is biologically active.

Resolvin mainly promotes the apoptosis of inflammatory cells and the clearance of apoptotic cells by increasing the phagocytic debris of macrophages and apoptotic PMNs, reducing the production of proinflammatory cytokines, reducing the expression of adhesion molecules, and reducing the infiltration of leukocytes and pain at the site of inflammation, which ultimately promotes the resolution of inflammation. Its related signalling pathways include NF-*κ*B, MAPK, and Caspase-3/9.

Chemerin chemokine-like receptor 1 (CMKLR1, also known as CHEMR23) of RvE1 is expressed in macrophages and dendritic cells. The high expression of IL-1*β*, IL-6, macrophage inflammatory proteins-1*α* and -*β*, and MCP-1 was inhibited through the interaction of RvE1 with CMKLR1. This attenuated TNF-*α*-mediated NF*κ*B activation inhibited neutrophil superoxide production, neutrophil infiltration, proinflammatory cytokine production, and enhanced macrophage activity. RvE1 can reduce the expression of CD18 on the surface of leukocytes, inhibit the flow of leukocytes in the blood vessel wall, and reduce leukocyte extravasation [43]. RvE1 can also bind to the receptor of LXA4 to upregulate the expression of related inflammation resolution genes, thereby reducing the inflammatory response of glial cells in a rat brain injury model [43]. RvE3 can strongly inhibit the inflammatory infiltration of neutrophils [44].

RvD1 also binds to LXA4 receptors ALX and GPR32, inhibiting inflammatory responses. RvD1 also attenuated TNF-*α*-mediated NF*κ*B activation and prevented inflammation amplification. RvD1 can also competitively inhibit the binding of LTB4 to its receptors in neutrophils, attenuate its activation of downstream signals, inhibit LTB4-induced neutrophil adhesion molecule expression, and limit neutrophil adhesion and infiltration. RvD1 exerts an anti-inflammatory effect through competitive inhibition. RvD2 can reduce the expression of TNF-*α*, IL-6, IL-1*β*, IL-23, and IL-1, regulate the production of NO, and regulate the expression of adhesion receptors on the surface of leukocytes [44]. AT-RvD1 and RvD3 can also bind to GPR32. In E. coli and S. aureus infections, RvD2 can limit the process of neutrophil infiltration and can enhance the process of bacterial clearance by phagocytes. In neural tissue, MaR1 and RvD1 can downregulate the severity of *β*-amyloid-induced inflammation. RvD2, through its receptor GPR18/DRV2, enhances phagocytosis of E. coli and apoptotic neutrophils in a protein kinase A- and STAT3-dependent manner [36].

PD1 is anti-inflammatory and inhibits the infiltration of leukocytes in the mice model of ischemic stroke, reduces airway eosinophil recruitment, reduces proinflammatory cytokine production, and reduces airway hyperresponsiveness in the mice model of asthma, accelerated neutrophil apoptosis and inflammation regression in the mice model of LPS-induced acute lung injury [45]. It can also promote the resolution of neuroinflammation and prevent the development of epilepsy [46]. BCL-XL and BCL-2 are antiapoptotic proteins. BAD and BAX are proapoptotic proteins. Regarding antiapoptosis, PD1 can upregulate the expression of BCL-XL and BCL-2 and downregulate the expression of BAD and BAX. Expression inhibits further expansion of inflammation by promoting clearance of CCR5 ligands. PD1 can also facilitate the process of macrophage phagocytosis of apoptotic neutrophils.

PDX, an isomer of PD1, can enhance the phagocytic function of macrophages. PDX also has anti-inflammatory effects by reducing the infiltration of neutrophils. In the mice model of postoperative ileus, lack of 12/15-LOX resulted in decreased PDX synthesis, increased neutrophil influx [47], and promoted inflammatory responses.

### 7.4. Product Maresins

DHA can generate 14S-Hp-DHA via 12-LOX, and this intermediate is catalyzed by soluble epoxide hydrolase (sEH) to generate Maresin 1 (MaR-1) and Maresin 2 (MaR-2) [48]. Maresins possess 22 carbon atoms and six double bonds and are also members of SPMs [15], which are synthesized by macrophages in the local inflammatory microenvironment.

Macrophages synthesize not only MaR1 but also transcellular synthesized in blood vessels by interacting with PMNs and platelets [49]. MaR1 can reduce the production of IL-1*β*, TNF-*α*, IL-6, and INF-*γ*, reduce the expression of ICAM-1, inhibit the infiltration of PMN, and reduce the manifestations of antiapoptotic proteins Mcl-1 and Bcl-1. MaR1 can promote the apoptosis of PMNs, increase the phagocytosis of pathogens and apoptotic PMNs by macrophages, and ultimately play an anti-inflammatory role. MaR2 can also reduce PMN infiltration and increase macrophage phagocytosis of pathogens and apoptotic neutrophils, but its effect is weaker than MaR-1 [50]. In neural tissue, MaR1 and RvD1 can also downregulate *β*-amyloid-induced inflammation and play a neuroprotective role [37].

### 7.5. SPMs

SPMs include maresins, lipoxins, protectins, and resolvins. In the inflammatory response, SPMs can inhibit neutrophil activation, reduce neutrophil accumulation in inflamed tissues, counteract proinflammatory cytokines, increase CCR5 expression in apoptotic cells, and enhance macrophage phagocytosis. SPMs help to quickly clear pathogens and repair injured tissue, thereby reducing the inflammatory response and promoting inflammation resolution.

In macrophages, SPMs trigger the shape changes of macrophages to prepare for the subsequent process of microbial phagocytosis and the process of apoptosis, enhance phagocytic function, and reduce proinflammatory cytokine production. In neutrophils, SPMs trigger the shape changes of leukocytes, limit the migration of neutrophils, inhibit neutrophil activation in tissues, reduce leukocyte adhesion, and promote the clearance of apoptotic neutrophils, thereby exerting a powerful anti-inflammatory effect. Natural killer cells (NK cells) express the lipoprotein A4 receptor, ALX. LXA4 binds to ALX to increase NK cell-mediated apoptosis of eosinophils and neutrophils, limit pathogen-mediated inflammatory responses, and promote the end of inflammation. NK cells can also express the receptor CMKLR1 of RvE1, which enhances the protective effect of RvE1. In the eosinophilic airway inflammation which induced by IL-33, the numbers of infiltrating eosinophils and type 2 innate lymphocytes (ILC2s) are increased in the airways, and both MaR1 and RvD1 can inhibit cytokine production by ILC2s [51]. ILC2s also express receptors for LXA4 and RvE1, which inhibit the release of proinflammatory cytokines from ILC2s. RvE1 reduces the production of IL-17. MaR1 binds TGF*β* and induces T cell formation. RvD1 can increase B cell antibody production [36].

## 8. Conclusion

Inflammation is related to the pathophysiological processes of many diseases. 12/15-LOX and its various metabolites produced by using different unsaturated fatty acids as substrates can participate in multiple inflammatory diseases by regulating the activity and function of immune cells. This effect is not only played through a single pathway and product but a complex metabolic regulatory network and the competitive inhibition of similar metabolic pathways or similar substrates. However, some anti-inflammatory and proinflammatory mechanisms are still unclear, and further research is needed to provide better guidance for clinical practice.

## Figures and Tables

**Figure 1:** Classification of polyunsaturated fatty acids.

**Figure 2:** Metabolic pathway of arachidonic acid. COX is cyclooxygenase. PGs are prostaglandins. CYP450 is cytochrome P450 monooxygenase. EETs are epoxyeicosatrienoic acids. LOX is lipoxygenase. LTs are leukotrienes. 12S-HpETE is 12S-hydroperoxy-eicosatetraenoic acid. PhGPx is phospholipid-hydroperoxide glutathione peroxidase. 12-HETE is 12-hydroxyeicosatetraenoic acid. HXA3 is hepoxilin A3. EH is epoxy hydrolase. TrXA3 is trioxilin A3.

**Figure 3:** Molecular structure formula of lipoxin. (a) shows the molecular structural formula of lipoxin A4 (LXA4). (b) shows the molecular structural formula of LXB4. (c) shows the molecular structural formula of their isomer 15-epimer-lipoxin A4 (15-epi-LXA4). (d) shows the molecular structure formula of 15-epi-LXB4.

**Figure 4:** Three ways of the generation of lipoxin. LTA4 is leukotriene A4. LXA4 is lipoxin A4.

**Figure 5:** The metabolic pathway of linoleic acid. HpODE is hydroperoxyctadecadienoic acid. HODE is a hydroxidecadienoic acid.

**Figure 6:** The production pathways of DHA, EPA, and AA. (a) shows the process of generating GLA and AA from linoleic acid. (b) shows the process of EPA and DHA generation by ALA. AA is arachidonic acid. GLA is *γ*-linolenic acid. ALA is *α*-linolenic acid. EPA is eicosapntemacnioc acid. DHA is docosahexaenoic acid.

**Figure 7:** Metabolic pathways of EPA and DHA. COX is cyclooxygenase. PGs are prostaglandins. LOX is lipoxygenase. LTs are leukotrienes. 12S-HpETE is 12S-hydroperoxy-eicosatetraenoic acid. 12-HEPE is 12-hydroxyeicosapentaenoic acid. HXB4 is hepoxilin B4. EH is epoxy hydrolase. TrXB4 is trioxilin B4. LXA5 is lipoxin A5. 14-HpDoHE is 14-hydroperoxydocosahexaenoic acid. MaR-1 is Maresin 1. 14-HDoHE is 14-hydroxydocosahexaenoic acid. 17S-Hp-DHA is 17S-hydroperoxy-docosahexaenoic acid. RvD1 is resolvin D1. PD1 is Protectin 1.

**Figure 8:** Different metabolites of AA and EPA catalyzed by the COX pathway and LOX pathway. (a) is the COX pathway. (b) is the LOX pathway. COX is cyclooxygenase. LOX is lipoxygenase. PG is prostaglandin. LT is leukotriene.

**Figure 9:** Molecular structure formula of resolvin (Rv) and protectin (PD). (a) shows the molecular structural formula of resolvin D1 (RvD1). (b) shows the molecular structural formula of resolvin E1(RvE1). (c) shows the molecular structural formula of Protectin 1 (PD1).

**Figure 10:** The generation of resolvin. COX is cyclooxygenase. LOX is lipoxygenase. RvD1 is resolvin D1. RvE1 is resolvin E1. AT is acetylated. 17S-Hp-DHA is 17S-hydroperoxy-docosahexaenoic acid.

## Data Availability

The data underlying the results presented in the study are available within the manuscript.
